The article "A Severity Score and Outcome Prediction in Patients that Suffered an Ischemic Stroke" was published in 2023. Journal: Emerg Med Int.

# A Severity Score and Outcome Prediction in Patients that Suffered an Ischemic Stroke

**DOI:** 10.1155/2023/5931502

**Published:** 2023-05-22

**Authors:** Corina Roman-Filip, Maria-Gabriela Catană (Vlădoiu), Mădălina Văleanu, Romeo-Gabriel Mihăilă

**Affiliations:** ^1^Neurology Department, Emergency County Clinical Hospital Sibiu, Corneliu Coposu bvd, Sibiu 550245, Romania; ^2^Faculty of Medicine, Lucian Blaga University of Sibiu, Izvorului Street, Sibiu 550169, Romania; ^3^Department of Medical Informatics and Biostatistics, University of Medicine and Pharmacy “Iuliu Haţieganu” Cluj-Napoca, 7 Horea Street, Cluj-Napoca 400174, Romania; ^4^Hematology Department, Emergency County Clinical Hospital Sibiu, Sibiu Corneliu Coposu bvd, 550245 Sibiu, Romania

## Abstract

**Background:**

Stroke is the main cause of disability and exitus worldwide. The prediction of mortality of this pathology represents a major challenge. More than that, the infection with the SARS-CoV-2 virus is a challenge for every clinician worldwide, and hypercoagulability is one of its biggest concerns that can lead to stroke.

**Objective:**

Our aim was to develop a severity stroke index for both SARS-CoV-2 stroke patients and noninfected stroke patients which we hope to be helpful in patient's management.

**Methods:**

We conducted a prospective study during January 2021–June 2021 which included 80 patients who suffered an ischemic stroke, 40 of which had both stroke and SARS-CoV-2 infection. We have established a panel of biomarkers including CRP, IL-6, fibrinogen, ESR, D-dimer, leucocytes, lymphocytes, and NLR and compared the results of our two cohorts.

**Results:**

SARS-CoV-2 stroke patients have experienced elevated levels of biomarkers that rise in inflammation such as hs-CRP, IL-6, and D-dimer, comparing to noninfected stroke patients. Also, the probability of exitus in SARS-CoV-2 patients is 4.2 times higher than in noninfected subjects. With regard to stroke severity, we have concluded that a NIHSS score higher than 15 points considerably influences the death rate, the probability of exitus being 9.16 times higher than in NIHSS score lower than 15.

**Conclusion:**

Based on our result, we have established a severity score index which includes NIHSS score, age, gender, the presence/absence of COVID-19 infection, and the following biomarkers: hs-PCR, IL-6, D-dimer, fibrinogen, and ESR, which can be used as a tool to guide patient's management.

## 1. Introduction

In 2019, SARS-CoV-2 infection was a challenge for every clinician worldwide. Almost three years since the pandemic began we know a lot more about the enemy we are fighting against, but we still have not figured out all the methods to prevent both the infection with this virus and especially the subsequent complications [1, 2]. One of the challenges that can appear in a patient that is infected with SARS-CoV-2 is the hypercoagulability that can lead to ischemic events, the most common being the stroke and myocardial infarction. A retrospective study that was conducted in Wuhan at the beginning of the pandemic concluded that 5% of the patients that were admitted to the hospital had a stroke with severe acute respiratory failure caused by an infection with SARS-CoV-2 virus. 90.9% of the subjects included in the study suffered an ischemic stroke, and 9.1% were reported to have an intracerebral hemorrhage [2, 3]. A case definition for COVID-19-related stroke was not sketched, but recent literature research that included subjects with and without SARS-CoV-2 infection and everyday experience supports the idea that between infection with SARS-CoV-2 and stroke could be a cause-effect association. It is clear that ischemic stroke was predominant, similar to the known epidemiology of cerebrovascular diseases. However, it was seen as a major increase in the cryptogenic etiology when TOAST classification was used [4, 5]. Studies have concluded that males were more affected and more often occluded large vessels are seen in patients without typical risk factors or symptoms of SARS-CoV-2 infection at stroke onset [1–4]. The most worrying is the fact that outcomes among stroke patients infected with SARS-CoV-2 seem worse than in stroke patients without SARS-CoV-2 infection; this being the reason why we give outmost importance to develop a prognostic risk score for patients who suffered a stroke, with or without SARS-CoV-2 infection [6].

## 2. Materials and Methods

### 2.1. Study Design

We conducted a prospective study during Jan 2021–June 2021 which included 80 patients who suffered an ischemic stroke, 40 of which had both stroke and SARS-CoV-2 infection. More exactly, the inclusion and exclusion criteria were stated, and the patients were surveilled while they were hospitalised.

Inclusion criteria are as follows:
  - Ischemic stroke in an adult subject that was admitted to the Emergency County Clinical Hospital Sibiu
  - Brain imaging describing an ischemic stroke by highlighting the lesion or its indirect signs
  - Ischemic stroke with onset <24 hours
  - For 40 patients, SARS-CoV-2 infection was confirmed by a RT-PCR test and characteristic symptoms were cough, fever, shortness of breath, and fatigue
  - Among the 40 patients, some patients were without SARS-CoV-2 infection and some patients were not vaccinated and were not infected at any time with SARS-CoV-2 virus and negative RT-PCR test result and no characteristic symptoms
Exclusion criteria for both groups are as follows:
  - Any medical pathology that can modify inflammatory markers: autoimmune disease, infections (other than SARS-CoV-2 infection), fever caused by a bacterial or viral infection other that SARS-CoV-2 infection, and oncological or hematological diseases (lymphomas, multiple myeloma, etc.)
  - Patients that have received treatment recently (in the last month) with corticosteroids or immunosuppressant medication
  - Patients with known myocardial infarction or myocarditis in the last 180 days
  - Patients who suffered a traumatic brain injury which was discovered during the neurological examination

It is important to mention that the Ethics Committee approved the study and all patients or the relatives empowered gave written informed consent to be included in the present study.

### 2.2. Blood Sample Collection and Biomarker Measurement

Blood samples were collected at hospital admission in the first 24 hours after the onset of the stroke. All blood samples were collected into EDTA (ethylenediaminetetraacetic) tubes. They were centrifuged at 1500 ×g for 15 min and were frozen at −80°C. Our biomarker panel included CRP, IL-6, fibrinogen, ESR, D-dimer, leucocytes, lymphocytes, and NLR. Biomarker measurement was performed by an ELISA device, according to the manufacturers' instructions. NLR was obtained by creating a ratio between neutrophils and lymphocytes. In terms of radiological biomarkers, the CT severity score has been calculated, the maximum value being 25 points.

### 2.3. Statistical Analysis

The database was maintained with the help of Microsoft Office Excel 2016. For the statistical analysis and data processing, we used the SPSS 25.0 (SPSS Inc, Chicago, USA) programme. The normal distribution of quantitative data was verified through the Kolmogorov–Smirnov test. The accepted error threshold was *α* = 0.05. To describe the continuous quantitative data normally distributed the average was used (standard deviation), and for the ones that did not have a Gaussian distribution, the median was used (quartile 1–quartile 3). In order to compare the median quantitative variables of two independent groups, we used Student's test (*t*-test) when the variables were normally distributed. The nonparametric tests, the Mann–Whitney and Kruskall–Wallis, were used to compare the averages of two independent groups in which there was an abnormal distribution. To compare the qualitative variables, the chi-squared and Fisher exact tests were used. The odds ratio (OD) and the trust interval associated (95% CI) according to the accepted error threshold were calculated. In order to determine the diagnostic value of some parameters, the ROC (receiver operating characteristic) curves were built and compared.

## 3. Results

A total of 80 patients with ischemic stroke were included in the study. Among them, 40 patients (50%) had SARS-CoV-2 infection and the other half being noninfected. The median age between these two groups of patients was similar: 70.25 for SARS-CoV-2 infected patients and 70.03 for noninfected patients. No significant differences in the gender distribution were noted in the noninfected group: 19 females (47.5%) versus 21 males (52.5%). With regard to SARS-CoV-2 patients, male sex is more prominent in this group: 15 females (37.5%) versus 25 males (62.5%). The intravenous thrombolytic medication (alteplase–rtPA) was administered in 6 out of 40 SARS-CoV-2 infected patients (15%) and 13 out of 40 noninfected patients (32.5%).

Comparing the two groups (infected versus noninfected), stroke patients associated with SARS-CoV-2 infection have experienced elevated levels of CRP (median, 34.97 [interquartile range, 8.71–75.35] versus 5.07 [2.31–8.38], *P* value <0.001), D-dimer (2405 [710.5–6226.98] versus 669 [478.2–1220], *P* value <0.001), and IL-6 (14.95 [8.7–29.78] versus (8.1 [7.3–9.3], *P* value <0.001) (Figures 1 and 2).

It was also observed that SARS-CoV-2 infection in stroke patients is significantly associated with exitus. Fifteen (37.5%) deaths occurred within the SARS-CoV-2 group of patients, comparing with the noninfected group where only five patients (12.5%) have died (*P* value <0.01). The probability of exitus in SARS-CoV-2 patients is 4.2 times higher compared with noninfected patients (OR = 4.2, 95% CI 1.35–13.065).

There is a strong correlation between the pulmonary CT scan severity score and the NIHSS (*r* = 0.742, *P* value <0.0001), increasing the latter determines an increase in the CT scan score. NIHSS is also a relevant indicator in the Severity Index Score and it is directly proportional to it. The univariate analysis shows that the following variables are significant for the Severity Index Score: NIHSS > 15 pts (it increases the probability of death by 25 times–OR = 25.242, 95% CI: 6.283–101.417), CRP, fibrinogen, ESR, D-dimer, NLR, and IL-6 levels (Figures 3 and 4).

Logistic regression shows that a NIHSS score higher than 15 points considerably influences the death rate, the probability of exitus in patients with NIHSS > 15 pts being 9.16 times higher than in patients with NIHSS < 15 pts (OR = 9.1674, 95% CI:. 1.723–48.762). The multivariate analysis suggests that the NIHSS score is correlated with fibrinogen and IL-6 levels so that these three variables influence the death rate at the same time (Figure 5).

## 4. Discussions

Our study describes the clinical outcome and the involvement of inflammation in patients with ischemic stroke and infected with SARS-CoV-2 compared with the control stroke patients. COVID-19 is a multisystem disease and behind its manifestations, there is a mutual pathological mechanism represented by a hyperinflammatory reaction and thrombosis [1, 2]. Furthermore, it is well-known that cerebral ischemia generates an inflammatory response both locally and in the peripheral circulation [2, 3].

Numerous studies have reported high levels of proinflammatory cytokines in the blood samples of the patients that were infected with SARS-CoV-2. Also, a meta-analysis of 16 retrospective studies showed that inflammatory biomarkers, such as IL-6, CRP, and ESR, were positively correlated with SARS-CoV-2 infection's severity [3–5]. Mehta et al., 2020, and Stebbing et al., 2020, also highlight the critical role of inflammatory biomarkers in progression of COVID-19 in patients [4, 5]. Similar to these results, our stroke patients, associated with SARS-CoV-2 infection, had been recorded much higher levels of inflammatory biomarkers, such as IL-6 (median value: 14.25 pg/ml vs. 8.1 pg/ml) and CRP (median value: median value: 34.97 mg/L vs. 5.07 mg/L), comparing to the noninfected stroke patients. No correlation was found between the results of laboratory tests and the onset of symptoms. This fact suggests that the biomarkers included in our study are correlated with the severity of the disease and has nothing to do with the time considered as the onset of the stroke. However, the role of inflammatory markers in keeping track of the severity of SARS-CoV-2 patients still remains controversial [3, 6–8].

IL-6 is secreted by activated T cells and also by macrophages. It has numerous proinflammatory and proatherogenic consequences. This interleukin leads to the triggering of the hepatocyte production of CRP and fibrinogen [6–9]. Increased levels of IL-6 have been frequently associated with poor outcome after ischemic stroke. Some studies have shown that elevated baseline levels of IL-6 are associated with risk of exitus [2, 7–9]. Also, it has been shown that IL-6 is an indicator that could predict mortality both one year and two years after ischemic stroke [2, 8–10]. Our study also shows that higher levels of IL-6 influence the death rate, alongside with the NIHSS score and high levels of fibrinogen. Measuring the IL-6 level could improve the decision of the therapeutic scheme. There are a high number of studies that report a favourable outcome from blocking IL-6 signaling in SARS-CoV-2 patients [7, 10–13]. Although this inflammatory biomarker is really useful, it is quite expensive and this makes it difficult to test on a regular basis.

CRP is a sensitive marker that is elevated as an acute-phase response in inflammation, tissue damage, and infection. Both stroke and SARS-CoV-2 infection cause elevation of CRP levels. Chet et al. reported higher levels of CRP in severe COVID-19 patients comparing to nonsevere patients [3, 13–15]. Our study indicates that IL-6 and CRP should be considered indicators of severity especially in COVID-19 stroke patients and also indicators of predictability of death.

The death rate in the COVID-19 group of patients was significantly higher than in the noninfected stroke group. A meta-analysis of 8 studies reported that ischemic stroke was identified to be considerably correlated with a higher risk of mortality in patients that suffered an ischemic stroke and were infected with SARS-CoV-2 [9, 15–17]. Similarly to this meta-analysis, our study shows that the probability of death in SARS-CoV-2 patients is 4.2 times higher compared with the control stroke group.

Ntaois et al. indicate that ischemic stroke patients infected with SARS-CoV-2 have substantially significant stroke severity according to the NIHSS score and a greater risk for severe disability and exitus compared with patients that were not infected with SARS-CoV-2 [2, 16–18]. The patients included in the study represent a subset of ischemic stroke subjects that were infected with SARS-CoV-2. The infection definitely provided a prothrombotic state that led to vascular occlusions and extensive strokes [10, 17–20]. Similar to the study by Ntaois et al., our study highlights that a NIHSS score >15 points is a significant indicator of severity and death, increasing the probability of exitus by 9.6 times.

Following our statistical analysis, we have obtained cut-off values for multiple indicators in both SARS-CoV-2 stroke patients and in noninfected stroke patients. Exceeding these values is causing deterioration in our patients. Based on that, we have created a severity index score which we hope to be helpful in managing our patients.

## 5. Conclusions

Based on our result, we have established a severity score index which includes the NIHSS score, age, gender, the presence/absence of COVID-19 infection, and the following biomarkers: hs-PCR, IL-6, D-dimer, fibrinogen, and ESR, which can be used as a tool to guide patient's management (Figure 6)

## Figures and Tables

**Figure 1:** ROC curve for SARS-CoV-2 stroke patients.

**Figure 2:** ROC curve for noninfected stroke patients.

**Figure 3:** Comparative levels of CRP between infected and noninfected patients.

**Figure 4:** Comparative levels of IL-6 between infected end noninfected patients.

**Figure 5:** Comparative levels of D-dimer between infected and noninfected patients.

**Figure 6:** Severity and outcome prediction score.

## Data Availability

The datasets used and/or analyzed during the current study are available from the corresponding author upon reasonable request.

## Abbreviations

hsCRP: High-sensitivity C-reactive protein
ESR: Erythrocyte sedimentation rate
IL6: Interleukin 6
NLR: Neutrophil to lymphocyte ratio
NIHSS: National Institutes of Health Stroke Scale
CT: Computed tomography.

## Additional Points

*Brief Summary.* This score is an important step forward for medical professionals who treat stroke patients. This score helps them so that they can easily follow the evolution of patients who have suffered a stroke and they can know what to expect regarding the prognosis.
